The article "SNAP-Tag Technology Optimized for Use in Entamoeba histolytica" was published in 2013. Journal: PLoS One.

# SNAP-Tag Technology Optimized for Use in *Entamoeba histolytica*

**DOI:** 10.1371/journal.pone.0083997

**Published:** 2013-12-31

**Authors:** Adam Sateriale, Nathan H. Roy, Christopher D. Huston

**Affiliations:** 1 University of Vermont Cellular, Molecular, and Biomedical Sciences Program, Burlington, Vermont, United States of America; 2 University of Vermont Microbiology and Molecular Genetics, Burlington, Vermont, United States of America; 3 University of Vermont Department of Medicine, Burlington, Vermont, United States of America; Centro de Investigacion y de Estudios Avanzados del Instituto Politecnico Nacional, Mexico

## Abstract

*Entamoeba histolytica* is a protozoan parasite responsible for invasive intestinal and extraintestinal amebiasis. The pathology of amebiasis is still poorly understood, which can be largely attributed to lack of molecular tools. Here we present the optimization of SNAP-tag technology via codon optimization specific for *E. histolytica*. The resultant SNAP protein is highly expressed in amebic trophozoites, and shows proper localization when tagged with an endoplasmic reticulum retention signal. We further demonstrate the capabilities of this system using super resolution microscopy, done for the first time in *E*. *histolytica.*

## Introduction

The protozoan parasite *Entamoeba histolytica* is a major cause of dysenteric disease throughout the developing world. Although most cases are asymptomatic, approximately 10% of cases develop into invasive amebiasis [1]. During invasive amebiasis trophozoites degrade the mucosal and epithelial layers of the host’s colon and migrate into the underlying tissue [2]–[4]. In rare cases there is formation of liver and even brain abscesses [1].

The underlying basis for an invasive *E. histolytica* infection is only beginning to become clear. It has recently been shown that a Q223R mutation in the human leptin receptor is associated with an increased infection rate [5]. This mutation is believed to decrease leptin-dependent STAT3-mediated activation, which renders host cells more susceptible to amebic cytotoxicity [6]. However, the mechanism of amebic cytotoxicity is still largely a mystery. It is known that *E. histolytica* secretes cysteine proteases and pore-forming peptides known as amoebapores [4], [7]–[11]. Yet host cell cytotoxicity appears to be largely apoptotic and contact dependent [12]–[14]. Understanding the basis of this observed pathology has been slow, mainly due to a lack of genetic and molecular tools.

Live cell imaging in *E. histolytica* is particularly challenging because the parasite is an obligate fermenter that can only withstand small amounts of molecular oxygen [15]. The most widely used tracking technique in the field is the expression of a green fluorescent protein (GFP) hybrid with the protein of interest. However, since GFP and its derivative protein tags rely on oxygen activation to achieve maximum fluorescence, it is necessary to express GFP-fusion proteins at high levels for visualization in *E. histolytica*, which can cause aberrant protein localization [16]. Here we present an alternative to GFP, a SNAP protein tag that has been optimized for the codon usage bias of *E. histolytica*. The SNAP protein is derived from the human DNA repair protein O6-alkylguanine-DNA alkyltransferase (hAGT), and acts irreversibly on O6-benzylguanine (BG) derivatives [17]. BG derivatives are amenable to a wide variety of labeling, from small molecules to fluorophores [18]. This allows for a greater versatility in label color and chemistry. The SNAP protein is not innately fluorescent, but rather becomes fluorescent when it binds irreversibly to fluorophore labeled O6-benzylguanine (BG) derivatives [17], [18]. This important aspect allows for the researcher to control the labeling process in both time and space.

## Materials and Methods

### Cell Culture

*Entamoeba histolytica* trophozoites, HM-1:IMSS strain grown in TYI-S-33 growth media, were used for all experiments [19]. During normal cell culture and antibiotic selection, amebas were grown in 15 mL glass tubes.

### SNAP Vector Construction

The backbone of the SNAP plasmid incorporates a previously described hygromycin selected tetracycline-inducible expression vector [20]. The codon optimized SNAP gene insert sequence is available as a supplementary data (Text S1). The oligos used to construct the upstream signal peptide and FLAG-tag were as follows: (forward) 5′-CATGAAATTATTATTATTAAATATCTTATTATTATGTTGTCTTGCAGATAAGCTAGATTATAAGGATGATGATGATAAGG-3′, (reverse) 5′- CTAGCCTTATCATCATCATCCTTATAATCTAGCTTATCTGCAAGACAACATAATAATAAGATATTTAATAATAATAATTTCATGGTAC-3′. The oligos used to construct the downstream KDEL amino acid endoplasmic retention signal were as follows: (forward) 5′-GATCTAAAGATGAGCTTTAACGATCGC-3′, (reverse) 5′-TCGAGCGATCGTTAAAGCTCATCTTTA-3′. The SNAP gene insert and all primers were produced by Integrated DNA Technologies, and all restriction enzymes used were produced by New England BioLabs. Trophozoites were transfected with 20 µg of plasmid DNA using the reagent Attractene (Qiagen) according to a previously described protocol [21]. Transfected amebas were selected using hygromycin, beginning with 1.5 µg/mL 24 hours following transfection. The concentration of hygromycin was slowly increased over the next 4 weeks to reach a final concentration of 15 µg/mL.

### Flow Cytometry and Western Blotting

Trophozoites were grown in 15 mL glass tubes, and then SNAP protein expression was induced for indicated times with 1 µg/mL tetracycline prior to prepping for flow cytometry. Tubes were placed on ice for 15 minutes to dislodge amebas, and then amebas were washed with phosphate buffered saline (PBS) and fixed with 4% paraformaldehyde for 20 minutes at room temperature. Amebas were permeabilized with 0.2% Triton-X, and then blocked for 30 minutes in 10% goat serum/5% bovine serum albumin in PBS. SNAP substrate (505-STAR (New England BioLabs)) was added to a final concentration of 5 µM, and amebas were incubated for 1 hr at room temperature. Trophozoites were washed 4 times with PBS, and then fluorescence was measured using a Beckman Coulter EPICS XL-MCL flow cytometer. Results represent two biological replicates from each time point, with 10,000 cells measured in each.

Amebas were grown in 15 mL glass tubes for immunoblotting, and received 1 µg/mL tetracycline 24 hours prior to harvest. Trophozoites were resuspended in cold lysis buffer (50 mM Tris-Cl, 300 mM NaCl, 1.0% Triton X-100) containing protease inhibitors (400 µM AEBSF, 200 µM EDTA, 60 nM aprotinin, 200 µM leupeptin, 2.8 µM E64, and 26 µM bestatin). 40 micrograms of protein from each sample was loaded into a 12% SDS-PAGE gel in reducing conditions. The gel was transferred to a PVDF membrane and blocked for 1 hour in Odyssey Blocking Buffer with 0.1% (v/v) Tween. Antibody to the SNAP protein (New England BioLabs) was used at 1∶1000, and labeled using IRDye 680 CW at 1∶5000. Infrared fluorescence was measured using an Odyssey LiCor CLx.

### Fluorescence Microscopy

For colocalization of the SNAP protein with native calreticulin, ameba were grown to mid-log phase in 15 mL glass tubes, and then induced with tetracycline for 24 hrs at a concentration of 1 µg/mL. Amebas were dislodged from these glass tubes and allowed to adhere to sterile glass coverslips for 30 minutes at 37°C. Cells were washed with PBS, and then fixed using 4% paraformaldehyde. Following fixation, amebas were again washed with PBS, and then blocked using 10% goat serum/5% bovine serum albumin in PBS. SNAP tagged substrate was used at 5 µM concentration for 1 hr. Calreticulin was visualized using a previously described scFv monoclonal antibody at 1 µg/mL [22]. Trophozoites were imaged using a Nikon Eclipse Ti2000 microscope with a 60× (1.4 NA) oil immersion objective. Images were taken using a Z-spacing of 0.267 µm, and then deconvolved using Autoquant X software (MediaCybernetics).

For live cell microscopy, trophozoites were grown to mid-log phase in 2 mL glass tubes, and then induced with tetracycline for 24 hrs at a concentration of 1 µg/mL. Following induction, SNAP substrate (TMR-STAR (New England BioLabs)) was added to a final concentration of 3 µM, and amebas were incubated at 37°C for 6 hrs. Media was then changed with new TYI-S-33 and labeled trophozoites were dislodged and moved to a 35 mm MatTek plate. Ameba were allowed to adhere for 30 minutes at 37°C, and then growth media was removed and replaced with PBS containing 1% low melting point agarose. Amebas were imaged using a Nikon Eclipse Ti2000 microscope with a 60×(1.4 NA) oil immersion objective and a heated stage (37°C). Images were taken using a Z-spacing of 0.500 µm, and then deconvolved using Autoquant X software (MediaCybernetics).

### STORM Microscopy

*Entamoeba histolytica* trophozoites were grown to mid-log phase in 2 mL glass tubes, and then induced with tetracycline for 24 hrs at a concentration of 1 µg/mL. Following induction, SNAP substrate (SNAP-Surface 647 New England BioLabs) was added to a final concentration of 5 µM, and ameba were incubated at 37°C for 6 hrs. Cells were washed with PBS, fixed using 4% paraformaldehyde, and again washed with PBS. Stochastic optical reconstruction microscopy (STORM) imaging was done as described previously, using a Nikon Eclipse Ti microscope base operating Nikon N-STORM software within NIS Elements (version AR 4.13.04) [23]. Image acquisition was performed using a 150 mW 647 nm laser in TIRF mode on continuous illumination. The STORM imaging buffer was composed of 50 mM Tris-HCl, 10 mM NaCl, 10% glucose, and 0.1 M cysteamine (Sigma). Buffer was supplemented with an enzymatic oxygen scavenging system using glucose oxidase (Sigma) and catalase (Sigma). 30,000 frames per image were collected at a rate of 50 Hz using a 100×PlanApo 1.45NA Nikon objective projected on an Andor iXon DU897 EMCCD camera. Single molecule fitting and image rendering was performed with N-STORM software within NIS Elements (version AR 4.13.04).

## Results

### Codon Optimized SNAP-tag Expression in *E. histolytica*

Our preliminary experiments of SNAP-tag protein expression in *E. histolytica* using the commercially available mammalian codon based DNA template proved unsuccessful (data not shown). Because the parasite has a highly AT rich genome, we hypothesized that altering the codons for the bias of *E. histolytica* might allow for increased SNAP-tag protein production. A new DNA sequence for the SNAP protein was constructed using synonymous codons reported to be overrepresented in *E. histolytica* genes with high expression [24]. Following codon optimization, the nucleotide composition of the SNAP-tag consisted of ∼55% AT, which more closely resembles that of the parasite genome, which is ∼75% AT (full sequence in Text S1) [15]. In order to test the expression and localization of the codon optimized SNAP-tag, we attached a KDEL localization signal specific for the endoplasmic reticulum, and used a tetracycline inducible vector for expression (Figure 1a). Tetracycline induction of SNAP protein expression, measured via flow cytometry, showed a peak in fluorescence at 24 hours that slowly tapered off (Figure 1b). The expression profile over time is in concordance with previously published data for other proteins expressed using this vector [20]. At 24 hours of tetracycline induction, SNAP protein expression was measured by quantitative infrared Western blot at approximately 76 times over background expression compared to lysate from trophozoites transfected with an empty vector control (Figure 1c). Visualization of the SNAP-tag in fixed trophozoites using a fluorescent O6-benzylguanine derivative together with antibody tagged calreticulin showed proper colocalization within the endoplasmic reticulum (Figure 2).

**Figure 1:** Tetracycline-regulated SNAP protein expression in *E. histolytica*. (A) Vector maps of EhSNAPspFLAG with and without the KDEL endoplasmic reticulum retention signal. (B) Time course of SNAP-tag protein expression induction using tetracycline, measured by flow cytometry. Times indicated in hours post addition of tetracycline. Values are mean and standard deviation for two experiments. (C) Western blot of trophozoite lysate from transfected cells induced with tetracycline for 24 hours. SNAP protein expression was measured to be approximately 76 times greater in trophozoites expressing SNAP-kdel compared to an empty vector control.

**Figure 2:** Colocalization of the SNAP-kdel protein with *E. histolytica* calreticulin. This ameba was fixed and labeled using a SNAP-Cell 505 Star reagent and anti-calreticulin (scale bar is 10 µm).

### Live Cell Imaging

The SNAP substrate was able to effectively cross the *Entamoeba* cell membrane in live trophozoites, allowing for real-time visualization of protein dynamics (Figure 3, and see Movie S1). Images here are taken using the cell permeable SNAP-Cell TMR-STAR reagent in TYI-S-33 amebic growth media, which can be visualized using a rhodamine filter set. The SNAP-Cell 505-Star reagent, which can be visualized using a fluorescein filter set, proved unsuccessful for live cell imaging due to the high amount of background fluorescence in the growth media (data not shown).

**Figure 3:** Live cell microscopy using the SNAP-tag. Trophozoites were labeled using a SNAP-Cell TMR Star reagent for 6 hours prior to microscopy (scale bar is 10 µm).

### STORM

One feature of the SNAP-tag system that particularly intrigued us was the ability to use the super resolution microscopy technique, stochastic optical reconstruction microscopy (STORM). STORM allows for the visualization of cellular structures at a spatial resolution below the diffraction limit of light [25]. This is accomplished through rapid imaging as fluorophores switch between on and off states. For each image, only small subsets of fluorophore molecules are visible, and thus the positions of individual molecules do not overlap, allowing for the precise determination of their location. Processing these images together allows for accurate mapping of many individual florescent molecules. However, the method typically requires direct labeling of a primary antibody with an appropriate fluorophore, which is not always practical in the *E. histolytica* system given the limited availability of quality antibodies. Because of the many fluorophores available, SNAP-tag fusion proteins are well suited to STORM imaging in either live or fixed cells with little optimization required. Here we present the first super resolution light microscopy imaging of *E. histolytica* (Figure 4). The enhanced spatial resolution allowed us to see the three-way bifurcation typical of the endoplasmic reticulum with a localization precision of ∼50 nm. The same image taken without STORM optic settings (widefield) showed the power of this method.

**Figure 4:** STORM imaging of an *E. histolytica* trophozoite. Super resolution microscopy of the amebic endoplasmic reticulum (ER) using a SNAP-tag protein with a KDEL ER retention signal. Inlayed boxes and arrows show the three way bifurcations that are characteristic of the ER, and the improved resolution that the STORM method provided (scale bar is 500 nm).

## Discussion

Here, we have presented a new method for protein localization in the parasitic protist *E. histolytica*. By optimizing the codon usage in the mammalian gene encoding a SNAP protein tag, *E. histolytica* trophozoites can now express the SNAP-tag, and expression can be controlled using available tetracycline-regulated expression plasmids. SNAP-tag fusion proteins can be detected in fixed or living trophozoites using a variety of commercially available reagents, and as one demonstration of new possibilities for *E. histolytica* researchers, we used the SNAP-tag to enable STORM for super resolution light microscopy in *E. histolytica* for the first time. However, we have only begun to scratch the surface of the SNAP-tag system capabilities.

SNAP substrates can be transiently applied, yet become covalently bound to their tagged protein of interest. These attributes make the SNAP-tag system ideal for pulse-chase experiments, whereby the trafficking dynamics of labeled proteins can be explored *in vitro* or *in vivo* [26]. Protein-protein interactions can be quantified using SNAP technology coupled with fluorescence resonance energy transfer (FRET) [27]. SNAP labeled proteins can be locally inactivated in living cells when coupled with chromophore-assisted laser inactivation (CALI) [28]. SNAP substrates can also be targeted to specific organelles, conjugated to biotin for pull-down experiments, or even used to immobilize tagged proteins onto printed structures [29], [30].

The SNAP-tag system represents a substantial improvement in the ability to track and image proteins in *E. histolytica*. The large variety of molecules that can be conjugated onto BG derivatives enables the adaptation and creation of new methods to study this protozoan parasite. We hope that these methods will enable the *E. histolytica* research community to better understand the pathology of amebiasis.

## Supporting Information

Text S1 ***E. histolytica*** **codon optimized SNAP protein sequence.**
(TXT)

Movie S1 ***E. histolytica*** **trophozoites expressing the SNAP protein with an endoplasmic reticulum localization signal.** SNAP protein was visualized using a SNAP-Cell TMR Star reagent (New England Biolabs). Shown at 3× normal speed.
(AVI)
